The article "Efficient drug delivery potential and antimicrobial activity of biocompatible hydrogels of dextrin/Na-alginate/PVA" was retracted in 2025. Reasons: unreliable results or conclusions; concerns about the authorship.

# Efficient drug delivery potential and antimicrobial activity of biocompatible hydrogels of dextrin/Na-alginate/PVA

**DOI:** 10.1016/j.heliyon.2024.e29854

**Published:** 2024-04-17

**Authors:** Arif Nazir, Mazhar Abbas, Faiza Kainat, Dure Najaf Iqbal, Farheen Aslam, Abida Kamal, Osama A. Mohammed, Kinza Zafar, Amal Abdullah Alrashidi, Samar Z. Alshawwa, Munawar Iqbal

**Affiliations:** a Department of Chemistry, The University of Lahore, Lahore, Pakistan; b Department of Basic Sciences, University of Veterinary and Animal Sciences, Lahore, (Jhang-Campus), Pakistan; c Department of Biotechnology, Lahore College for Women University, Lahore, Pakistan; d Department of Chemistry, University of Agriculture, Faisalabad, Pakistan; e Department of Pharmacology, College of Medicine, University of Bisha, Bisha, 61922, Saudi Arabia; f Medical Unit#2, Lahore General Hospital, 54000, Lahore, Pakistan; g Department of Pharmaceutical Sciences, College of Pharmacy, Princess Nourah bint Abdulrahman University, P.O. Box 84428, Riyadh, 11671, Saudi Arabia; h Department of Chemistry, Division of Science and Technology, University of Education, Lahore, Pakistan

**Keywords:** Hydrogels, Polymers, Biocompatible, Antibacterial activity, Biodegradation, Cytotoxicity, Drug delivery

## Abstract

Ceftriaxone sodium belongs to the third-generation cephalosporin group and is used intramuscular and intravenous route as a broad-spectrum antibiotic. This research aims to prepare biocompatible hydrogels for targeted delivery of ceftriaxone sodium by parental route. Different proportions of polymers (natural and synthetic) in the presence of cross-linker were synthesized by solvent casting method. Ceftriaxone sodium was loaded in hydrogels in different concentrations and its drug release behavior was evaluated along with swelling and biodegradation analysis. The characterization of hydrogel was done by scanning electron microscopy (SEM) and Fourier transform infrared (FTIR) to analyze surface morphology and functional groups involved in the formation of dextrin/Na-alginate/PVA hydrogels loaded with the drug. Thermogravimetric analysis (TGA) was confirmed by thermal stability and degradation pattern of loaded and unloaded hydrogels. The drug-loaded samples presented promising antimicrobial activity against *S. aureus* and *P. multocida* and their cytotoxic nature was also studied. Drug release analysis using simulated intestinal fluid (SIF) and phosphate buffer saline(PBS) for the circulatory system shows the consistent release of the drug. The findings unveiled the development of a biocompatible and innovative hydrogel, which has potential advantages for biomedical application, particularly in enhancing the therapeutic efficacy of ceftriaxone sodium drug.

The article "Efficient drug delivery potential and antimicrobial activity of biocompatible hydrogels of dextrin/Na-alginate/PVA" was retracted in 2025. Reasons: unreliable results or conclusions; concerns about the authorship.

## 1 Introduction

Hydrogels belong to a class of three-dimensional and moisturized polymeric networks. Hydrophilic polymer chains join to form hydrogels and these chains may be natural or artificially synthesized. The structural stability of hydrogel relies on cross-links developed by chemical and physical bonds among the polymer chains [[1], [2], [3], [4]]. Hydrogels offer advanced chances to develop various clinical uses such as drug delivery systems, scaffold products to arrange cells into a 3D network, cell replacements, wound dressings and immobilization of proteins and cells, among others. the medical benefits of hydrogels are increasing, substantial efforts have been made to create new hydrogels from a range of artificial and natural materials [[5], [6], [7]].

Drug delivery is the targeted introduction of pharmaceutical substances into organisms to achieve therapeutic effects. It involves modifying drug properties using excipients, carriers, and medical devices to enhance efficacy. Combining drugs with hydrophobic molecules can expand their applications and effectiveness [[8], [9], [10], [11], [12]]. Conventional drug delivery methods include oral, parenteral, topical, rectal and inhalation routes [13]. These methods enhance drug efficacy, regulate drug release, and provide sustained therapeutic effects. They optimize pharmacological effects, ensure targeted delivery to specific cells, and control biodistribution and pharmacokinetics for improved efficacy [[14], [15], [16], [17]]. Novel drug delivery systems offer enhanced bioavailability and solubility, sustained release profiles, improved pharmacokinetics, increased patient adherence to medication regimens, higher drug efficacy at lower doses, reduced adverse effects, and enhanced pharmacological activity. They also improve macrophage circulation, minimize chemical degradation, and provide other benefits [18,19].

Targeted drug delivery involves delivering medication to a specific site. It bypasses host defenses to reach the intended location and achieve the desired pharmacological action with minimal side effects [20,21]. These systems aim to enhance drug effectiveness, reduce adverse effects, and improve therapeutic index [22]. They can lead to increased therapeutic activity, decreased dosage requirements, and elimination of special drug administration methods [23]. Developing targeted drug delivery to specific tissues, such as heart cells, is crucial for future regenerative medicine. Passive targeting occurs naturally in the body, with neurotransmitters, growth factors, and hormones directly targeting sense organs. This can be applied to drugs through physical and physiochemical mechanisms, known as passive targeting [24]. Intracellular drug delivery involves endocytosis for drug entry into targeted tissues, such as sensory organs. Ideal drug carriers should be harmless, biocompatible, non-immunogenic, biodegradable, and recognized by the host defense system [25]. Liposomes are commonly used for sustained drug release [26]. Antibiotics inhibit microbial growth, with ceftriaxone sodium belonging to the cephalosporin group effective against gram-positive and negative bacteria. Ceftriaxone was discovered in 1978 and approved for clinical use in 1982 [25].

The article "Efficient drug delivery potential and antimicrobial activity of biocompatible hydrogels of dextrin/Na-alginate/PVA" was retracted in 2025. Reasons: unreliable results or conclusions; concerns about the authorship.

Hydrogel preparation involves the use of polymers and crosslinkers, which are essential for maintaining the hydrogels' mechanical characteristics, structural integrity, and drug-release behavior. Polymers provide the matrix for drug encapsulation and are the structural backbone of hydrogel networks. They ascertain the hydrogel's general physical and chemical characteristics, such as its swelling behavior, biocompatibility, and biodegradability. Various polymer types can be chosen according to their unique properties and suitability for the intended use. For instance, while synthetic polymers like polyvinyl alcohol (PVA) and polyethylene glycol (PEG) offer tunable mechanical properties and controlled drug release, natural polymers like alginate and chitosan offer biocompatibility and ease of gelation [27]. Crosslinkers are molecules that create a network structure within the hydrogel by joining polymer chains together. They are essential in regulating the hydrogel's mechanical strength, stability, and porosity. The hydrogel's swelling behavior and drug release kinetics are directly affected by the crosslinking density. Drug delivery applications can customize the hydrogel's properties to meet specific needs by varying the crosslinker type and concentration. For natural polymers, glutaraldehyde, genipin, and calcium ions are frequently utilized crosslinkers; for synthetic polymers, N,N'-methylenebisacrylamide (MBA) is used. Therefore, to prepare hydrogels with the necessary structural and functional qualities for efficient drug delivery applications, polymers and crosslinkers are crucial ingredients. To design hydrogels with desired properties like mechanical stability, controlled drug release, and biocompatibility, these components must be carefully chosen and optimized [28].

The objective of this study was to develop a biocompatible hydrogel composed of dextrin, sodium alginate, and polyvinyl alcohol (PVA) for delivering ceftriaxone sodium. The synthesized hydrogel was characterized to assess its physical and chemical properties. Drug release potential, biodegradation and swelling behavior of the hydrogel were also evaluated to understand its controlled release mechanism and responsiveness to aqueous environments. The aim is to develop an effective drug delivery system for optimizing the therapeutic efficacy of ceftriaxone sodium.

The article "Efficient drug delivery potential and antimicrobial activity of biocompatible hydrogels of dextrin/Na-alginate/PVA" was retracted in 2025. Reasons: unreliable results or conclusions; concerns about the authorship.

## 2 Material and methods

### 2.1 Chemicals and reagents

For the synthesis of hydrogels following chemicals and reagents were used, i.e., dextrin (from corn, type, powder, MW: 564.4 g/mole), sodium alginate (MW: 35000 g/mol) and Ceftriaxone sodium drug (C_18_H_16_N_8_Na_2_O_7_S_3_, MW: 661.60 g/mol), which were obtained from Sigma Aldrich. A polymer as well as binder i.e., polyvinyl alcohol (type of 25–98, 88–90% hydrolyzed, MW: 44.053 g/mol, polymerization degree of 2040±60, and alcoholysis degree of 98.9%), glutaraldehyde (MW: 100.12 g/mole, density: 1.07 g/cm³) cross-linker were also provided by Sinopharm Chemical Reagent Co., Ltd. All solutions were prepared using distilled water.

### 2.2 Preparation of hydrogels

By changing concentrations of polyvinyl alcohol (PVA) and sodium alginate (AG) with a fixed amount of dextrin (D) and glutaraldehyde (G), blended samples were prepared. Dissolution casting method was used to synthesize these blended films.

#### 2.2.1 DSAPG#1 sample

For the preparation of the DSAPG#1 sample, a beaker was filled with 40 mL distilled water and placed on a hot plate. Dextrin 0.4g (D) was weighed separately and added in the hot water, (Table 1). Dextrin was added in 3 batches to make a homogenous solution. A magnetic stirrer was used for homogeneous solution preparation. The solution was continuously heated, blended and stirred until no crystal was left. Temperature was monitored continuously and kept constant at 80 °C. After 40 min, the solution was homogenized. In a separate beaker, 0.2g of PVA (P) was dissolved in 20 mL of H_2_O with heating at 90 °C.

**Table 1:** Percentage composition of different blends of hydrogels.

Sr. #	Sample	Dextrin (g)	Na-alginate (g)	**PVA (g)**	**Glutaraldehyde (mL)**
**1**	DSAPG#1	0.4	0.3	0.2	0.1
**2**	DSAPG#2	0.4	0.3	0.3	0
**3**	DSAPG#3	0.4	0.4	0.1	0.1
**4**	DSAPG#4	0.4	0.4	0.3	0.1
**5**	DSAPG#5	0.4	0.4	0.2	0.1
**Drug loaded hydrogel films**					
**1**	CTX10	0.4	0.3	0.2	0.1
**2**	CTX25	0.4	0.3	0.2	0.1
**3**	CTX50	0.4	0.3	0.2	0.1

Another beaker was used to prepare 0.3g of sodium alginate solution in 30 mL of H_2_O. The above mixtures were suspended in the sodium alginate (SA) solution, blended and stirred with 0.1 mL of glutaraldehyde (G) at the same temperature for 2 h, till the volume of the mixture was reduced to one-third of the original volume. After complete blending, it was poured into the sterilized petri plates and dried for 24 h in a drying oven at 60 °C. Resultantly, a light yellow and flexible hydrogel film was formed. Then the hydrogel is subjected to air drying for 15 min till complete drying and removed carefully from molds placed in tight bags and subjected to characterization and analysis.

The article "Efficient drug delivery potential and antimicrobial activity of biocompatible hydrogels of dextrin/Na-alginate/PVA" was retracted in 2025. Reasons: unreliable results or conclusions; concerns about the authorship.

#### 2.2.2 DSAPG#2 sample

Dextrin (0.4 g) was dissolved in 40 mL of distilled water and heated at 80 ^°^C on a hot plate with continuous stirring for 40 min. In a separate beaker, 0.3g of PVA was dissolved into 30 mL of H_2_O with heating at 90 °C. Using a new beaker 0.3g of sodium alginate solution in 30 mL of H_2_O was prepared. Then, the above mixture was suspended in sodium alginate solution with constant stirring for 1 h. After complete blending, transferred into petri plates and placed in a drying oven at 60 °C for 24 h resultantly, a sticky and yellow-colored film was formed. Then, the hydrogel was removed from the petri plate and placed in an air-tight bag. Next batches (DSAPG#3, DSAPG#4 & DSAPG#5) are also fabricated via a similar technique just by changing the concentrations of polymers with constant dextrin and glutaraldehyde amounts.

### 2.3 Preparation of drug-loaded samples

The drug is loaded in DSAPG#1 with the same composition of dextrin (D), sodium alginate (SA), glutaraldehyde (G) and polyvinyl alcohol (PVA) as mentioned above. In a separate beaker, 10 mg of ceftriaxone sodium drug (CTX) was added to the prepared solution with constant stirring and heated at 50–60 °C for 1 h. After complete blending, poured into petri plate and dried at 60 °C for 24h. Resultantly, a transparent hydrogel (membrane) was obtained after loading the ceftriaxone sodium. Similarly, samples with 25 mg and 50 mg were prepared with the same method (Fig. 1).

**Fig. 1:** Physical appearance of synthesized various blends of hydrogels (DSAPG#1 contains dextrin 0.4 g, Na-alginate 0.3 g, PVA 0.2 g and glutaraldehyde 0.1 mL, DSAPG#2 contains dextrin 0.4 g, Na-alginate 0.3 g, PVA 0.3 g and glutaraldehyde 0.0 mL, DSAPG#3 contains dextrin 0.4 g, Na-alginate 0.4 g, PVA 0.1 g and glutaraldehyde 0.1 mL, DSAPG#4 contains dextrin 0.4 g, Na-alginate 0.4 g, PVA 0.3 g and glutaraldehyde 0.1 mL, CTX25 (25 mg drug) contains dextrin 0.4 g, Na-alginate 0.3 g, PVA 0.2 g and glutaraldehyde 0.1 mL, and CTX50 (50 mg drug) contains dextrin 0.4 g, Na-alginate 0.3 g, PVA 0.2 g and glutaraldehyde 0.1 mL).

### 2.4 Characterizations

The prepared hydrogels were characterized by different techniques. The hydrogel samples were characterized using FTIR, SEM, TGA and UV–visible techniques. The analysis of samples was done for functional group identification presents in the polymer and blended members. FTIR analysis of the prepared samples was accomplished using IR instrument ALPHA II having wavenumber 4000-680 cm^−1^ with resolution 16 and background scans are 10. The SEM is a type of characterization performed to recognize the surface morphology of the material. For this analysis, synthesized samples were assayed through FEI Nova NanoSEM 450. Different magnifications ranging from 100kx to 500kx were used to examine the surface morphology.

The article "Efficient drug delivery potential and antimicrobial activity of biocompatible hydrogels of dextrin/Na-alginate/PVA" was retracted in 2025. Reasons: unreliable results or conclusions; concerns about the authorship.

Light transmittance is a useful feature for hydrogel during disease-curing applications [29]. UV–Vis. light is allowed to interplay with the sample and then the transmittance and absorption of radiation are recorded. Thermogravimetric analysis is a thermal analysis in which the weight loss of a specimen can be measured with temperature. This measurement gives information about physical and chemical phenomenon, physically involves phase transitions, adsorption and desorption, while chemical phenomena include solid-gas interactions (e.g., oxidation or reduction) chemisorption and thermal degradation. The results were recorded with TA Universal Analysis 2000 Software.

### 2.5 Swelling behavior

The swelling properties of unloaded DSAPG and CTX-loaded samples were observed to measure the swelling percentage that plays the main role in attaining the release behavior of the drug and entrapment of the hydrogel [30]. The swelling capability of hydrogels was estimated in different buffer solutions and distilled water as a function of time. For this, a disk of precisely measured hydrogel was submerged in the respective media. After a stipulated period, the solvent was removed and the weight change was measured. This procedure was continued to achieve the constant weight. The swelling ratio was measured using Eq. (1), Where, W_s_ = Swollen hydrogel’s weight and W_d_ = dry hydrogel’s weight [31].

(1) $$\text{Swelling}\;\text{ratio}=\frac{Ws-Wd}{Wd}$$

### 2.6 Biodegradation study of the hydrogels

Phosphate-buffered saline (PBS) solution was used to submerge 50 mg of hydrogel samples to examine them *in vitro* biodegradation properties. We carefully tracked the hydrogels' weight loss throughout one, three, and six days. The hydrogel samples were then cautiously taken out from the PBS solution at the predetermined intervals, and any weight loss was carefully noted. The hydrogels in the PBS solution underwent a biodegradation process, which was indicated by the weight loss that was seen over time. This method gave important insights into the hydrogel formulations' stability and kinetics of degradation in physiological settings. A thorough grasp of the hydrogel's biocompatibility and potential use in biomedical applications could be obtained by measuring weight loss at various intervals to systematically analyze the temporal evolution of the biodegradation process. This arrangement made it possible to evaluate the *in-vitro* biodegradation behavior of hydrogels in detail, which helped to clarify their breakdown processes and direct future optimization for specific biomedical applications.

The article "Efficient drug delivery potential and antimicrobial activity of biocompatible hydrogels of dextrin/Na-alginate/PVA" was retracted in 2025. Reasons: unreliable results or conclusions; concerns about the authorship.

### 2.7 Antibacterial assay

For the antibacterial potential of (CTX25, CTX50) a panel of gram-positive and gram-negative strains (*Proteus vulgaris, Staphylococcus aureus, Pasteurella multocida* and *Escherichia coli*) was used by agar well diffusion method. A nutrient agar medium was used to sustain the culture medium of bacterial strains. A fresh bacterial culture of each strain 1.2 × 10^8^ CFU/mL was used in this assay. For this, a 10 mg hydrogel having CTX25 and CTX50 were dipped in 1 ml sterilized distilled water. A 20 mL of nutrient agar was added to each sterilized petri plate and 100 μL of fresh bacterial culture was added to each petri plate, mix it well for equal distribution and then left the plates for solidification. Using the sterilized method, wells were induced in each petri plate and 100 μL of hydrogel sample (CTX25, CTX50), along with control (ciprofloxacin 1 mg/mL), were transferred into each well and left the petri plates for 10 min in sterilization condition and then incubate them at 37 °C for 24 h. The sample indicating antibacterial potential inhibits the bacterial growth and clear zone was documented using a zone reader and reported in mm (millimeters) [32].

### 2.8 Drug release analysis

For the oral route of drug administration, the main objective is to prevent it from gastric fluid (pH∼1–2). Because major absorption of the drug takes place in the small intestine having pH∼6.8 and is transported to the site of infection by the circulatory system (pH∼7.4). To determine *in-vitro* sustainable drug (ceftriaxone sodium**)** release, the prepared samples were loaded with CTX25 and CTX50 and their release was monitored in PBS and SIF medium. The different buffer solution was prepared, i.e., following salts, NaCl (8 g), KCl (0.2 g), Na_2_HPO_4_ (1.44 g), KH_2_PO_4_ (0.24 g) with given concentration was used for phosphate buffered saline (PBS) preparation and to maintain its (pH∼7.4), few drops of hydrochloric acid (HCL) was used and finally, volume was maintained 1000 mL using distilled water [39]. For simulated intestinal fluid (SIF) preparation, the following solution was mixed, i.e., 250 mL solution of KH_2_PO_4_ (0.2 M) and 118 mL solution of NaOH (0.2 M) for the preparation of (pH ∼6.8) and distilled water was used to achieve the desired volume [40].

The article "Efficient drug delivery potential and antimicrobial activity of biocompatible hydrogels of dextrin/Na-alginate/PVA" was retracted in 2025. Reasons: unreliable results or conclusions; concerns about the authorship.

### 2.9 Hemolytic assay

Cytotoxicity of CTX25 and CTX50 was measured against *in-vitro* red blood cells (RBCs) with slight modification [33]. In this method, fresh human blood (4 mL) was collected and transferred into a pre-sterilized 15 mL falcon tube having heparin (a few drops) to avoid blood coagulation and suspended in isotonic phosphate buffer saline (PBS-pH 7.4) to avoid cell lysis. The content was centrifuged at 950*×g* for 10 min. The supernatant was poured off and RBCs were washed three times with 5 mL of chilled (4 °C) sterile isotonic phosphate buffer saline (PBS) solution, adjusted to pH∼7.4. The washed RBCs were suspended in the 20 mL isotonic phosphate buffer saline and cell counts; 4.068 × 10^6^/μL were maintained for hemolytic/cytotoxicity assay. A 10 mg of loaded hydrogel of (CTX25 and CTX50) was dipped in 1mLwater and 50 μL stock solutions containing ceftriaxone sodium was treated with 175 μL red blood cells (RBCs) suspended in phosphate buffer saline. The entire reaction mixture was incubated for 30 min at 37 °C. After the first 10 min of incubation, the mixture was agitated. Following the completion of the incubation period, the tubes were immediately placed on ice for 5 min before being centrifuged for 5 min at 1310×*g*. Following centrifugation, 100 μL of supernatant was carefully removed from each tube and diluted with 900 μL of chilled Phosphate buffer saline (PBS). It is worth noting that all eppendorf tubes were kept on ice after dilution to reduce the possibility of mechanical blood lysis. Following that, 200 μL of the mixture from each eppendorf tube was dispensed into the corresponding 96-well plate. A solution containing 0.1 % Triton X-100 was used as a positive control in each assay, while phosphate-buffered saline (PBS) was used as a negative control. The absorbance of the samples was measured using a BioTek Quant microplate reader (BioTek, Winooski, VT, USA) at a wavelength of 576 nm. The percentage of lysis was calculated using the relationship depicted in Eq. (2) to determine the extent of RBC lysis.

(2) $$\text{Lysis}\;\text{of}\;\text{RBCs}\;\left(\%\right)=\frac{\text{Absorbance}\;\text{of}\;\text{sample}}{\text{Absorbance}\;\text{of}\;\text{Triton}\;\left(X-100\right)}\times 100$$

## 3 Results and discussion

### 3.1 Functional group analysis

It is a characterization technique used for chemical classification and to identify the different functional groups and the response is depicted in Fig. 2. These results are collected in wavenumber units (cm^−1^). FTIR spectra of DSAPG#1 displayed a distinguishing wide-ranging band of O–H *str.* at 3220-3400 cm^−1^, an accurate peak of C–H stretching observed at 2923.51 cm^−1^, a distinctive peak related to C=O stretching at 1602.28 cm^−1^ (due to resonance of carboxylate ion), because of CH_2_ *bending,* a strong absorption presented at 1411.93 cm^−1^ and due to C–O–C str. vibration, a broad peak recorded at 1077 cm^−1^. However, in DSAPG#2, DSAPG#3, DSAPG#4 and DSAPG#5, there were variations in values which were correlated with the difference in concentration of ingredients in the prepared sample of hydrogels. The IR spectra of DSAPG#2, DSAPG#3, DSAPG#4 and DSAPG#5, exhibited distinctive absorption of O–H str. at 3220-3400 cm^−1^ an extensive band, C–H *str*. at 2500-3000 cm^−1^, C=O *str*. at 1400-1600 cm^−1^, C–O–C str. at 1077 cm^−1^, ether wide absorption took place at C–O *str*. at 1000-1020 cm^−1^ and due to CH_2_ bending a broad peak detected at 1300-1500 cm^−1^. Table 2 represents the ranges of absorption peaks observed in the prepared hydrogel membranes and the FTIR of individual SA and PVA are depicted in Figs. S1–S2, respectively. A potent analytical method for examining the chemical makeup and structure of hydrogels made of polyvinyl alcohol (PVA), sodium alginate, and dextrin is FTIR spectroscopy. The hydrogen bonding interactions between the hydroxyl groups in dextrin, sodium alginate, and PVA molecules are examples of the physical and chemical interactions that can be investigated using FTIR analysis. Hydrogen bond formation within the hydrogel matrix can be indicated by changes in the position and intensity of the hydroxyl group absorption bands in the FTIR spectrum. Furthermore, interactions between the PVA, sodium alginate, and dextrin polymer chains within the hydrogel matrix are conceivable. A physical interaction like polymer chain entanglement or a chemical interaction like crosslinking reactions can be indicated by changes in the absorption bands that correspond to particular functional groups in each polymer. In the hydrogel matrix, chemical crosslinking reactions can also take place. As an illustration, consider the emergence of new absorption bands or changes in absorption peaks linked to functional groups that are involved in crosslinking reactions (e.g., PVA or sodium alginate reacting with the aldehyde groups in dextrin). When comparing the hydrogel to the functional groups found in dextrin, sodium alginate, and PVA molecules, the hydrogels' interactions are also revealed. Changes in the hydrogel's hydration state or water-binding capacity may be indicated by variations in the position or intensity of the absorption bands that correspond to water molecules.

The article "Efficient drug delivery potential and antimicrobial activity of biocompatible hydrogels of dextrin/Na-alginate/PVA" was retracted in 2025. Reasons: unreliable results or conclusions; concerns about the authorship.

**Fig. 2:** FTIR spectra of synthesized various blends of hydrogels (unloaded and loaded with Ceftriaxone sodium drug).

**Table 2:** Vibrational absorption bands in IR spectra in different blends of hydrogels.

Fuctional groups	DSAPG#1 (cm^−1^)	DSAPG#2 (cm^−1^)	DSAPG#3 (cm^−1^)	DSAPG#4 (cm^−1^)	DSAPG#5 (cm^−1^)
O–H *str.*	3280.01	3259.54	3255.05	3271.03	3262.88
C–H *str*.	2923.51	2921.68	–	2921.89	2921.02
C=O *str*.	1602.28	1606.05^1^	1631.66	1607.25	1600.66
CH_2_*ben.*	1411.93	1414.58	1397.14	1416.07	1412.35
C–O *str* Carboxylic acid	–	1241.66	–	1245.51	1248.75
C–O–C *str.*	1077.34	1077.22	–	1076.81	1077.96
C–O *str.*	1018	1015	–	1015.99	1020.07

### 3.2 Surface morphology

To analyze the surface morphology of the prepared sample, a scanning electron microscope was employed [34]. The surface morphology of hydrogels composed of dextrin, sodium alginate, and polyvinyl alcohol (PVA) can be analyzed using scanning electron microscopy (SEM). SEM analysis allows for the visualization of surface features such as pores, channels, and surface roughness. The SEM analysis was performed of drug-unloaded (D/Na-Alg/PVA) and drug-loaded samples (D/Na-Alg/PVA/CTX) to evaluate the difference between both samples, which is useful to understand the effect of drug loading on the morphology of the hydrogel. The SEM images of the prepared hydrogel (unloaded) revealed the formation of a rough surface, indicating less crosslinking within the structure of hydrogel, which is promising to facilitate the absorption of water into the hydrogel matrix. The SEM analysis also revealed the formation of loose packing and spaces in the structure of hydrogels (Fig. 3ab). On the other hand, the drug-loaded sample (DSAPG#1) surface is changed slightly, which is due to the compactness of the drug with the structure of hydrogel and space in the structure of hydrogel are still visible. These spaces in the structure of hydrogel are useful to enter the water inside of the hydrogel and sustainably release the drug. In the drug-loaded hydrogel sample, the structure is neither compact nor loosely packed, which is ideal for drug loading and release when these are employed for drug delivery. These loose packing and the presence of spaces in the structure of prepared hydrogel revealed to be the source of water pervasion zones and interconnecting areas for ionic interaction, temperature sensitivity and pH. So, these blends show their hydrophilicity and swelling properties [35]. The presence of crosslinked alginate/PVA in the dextrin backbone caused the emergence of agglomerates with crevices, through which medium penetration is possible via crevices at the surface structure [36]. These images verified that the synthesized hydrogel has an irregular and porous structure, which favors the drug loading efficiency. When the drug was diffused into the sample DSAPG#1, a regular morphology was observed in the loaded CTX50 sample. It may arise from molecular interactions, such as hydrogen bonding between the percolated polymeric network and the drug during the drug encapsulation into the hydrogel system. The 50 mg ceftriaxone sodium loaded sample (CTX50) showed a clear difference with the unique sandy rose ontogeny of alginate-ceftriaxone sodium [37], which specified that sodium alginate takes effect as a dispersant of the drug and the drug has been completely dispersed on the surface of the hydrogel. The interface between the drug and hydrogel is entirely physical. The pores and holes present in the unloaded DSAPG#1 were filled with the drug ceftriaxone sodium and it has made the hydrogels beneficial for drug delivery loading and its subsequent delivery to the target. UV–vis spectra of dextrin, alginate, PVA and ceftriaxone sodium (DSAPG#1) were performed in the 200–800 nm range and the response is depicted in Fig. 4.

The article "Efficient drug delivery potential and antimicrobial activity of biocompatible hydrogels of dextrin/Na-alginate/PVA" was retracted in 2025. Reasons: unreliable results or conclusions; concerns about the authorship.

**Fig. 3:** Surface morphology of (a) DSAPG#1 sample and (b) DSAPG#1 drug (CTX50) loaded.

**Fig. 4:** UV–visible analysis of the DSAPG#1 drug loaded (CTX50) samples in PBS media (pH 7.4).

### 3.3 Thermogravimetric analysis

Thermogravimetric analysis (TGA) of dextrin/Na-alginate/PVA hydrogel provides valuable information about its thermal stability and degradation behavior [38]. The initial weight loss that was noted in the dextrin/Na-alginate/PVA hydrogels with and without drugs was described as the evaporation of bound water molecules, hydrogen-bonded water molecules, and moisture. This phenomenon happened as a result of the hydrogel matrix's high absorption capacity, which was specifically impacted by the presence of polyvinyl alcohol (PVA), sodium alginate, and dextrin. The drug-loaded and unloaded hydrogels underwent different degradation steps during this initial stage, indicating differences in their capacities to absorb water (Fig. 5). The subsequent stage of weight loss was ascribed to the breakdown of linkages within the dextrin/Na-alginate/PVA blends and the disruption of interactions between the various components of the hydrogel matrix. This degradation step denotes the disintegration of molecular interactions and chemical bonds in the hydrogel structure, which may have been impacted by the drug molecule present in the matrix. Ultimately, the breakdown of the polymer chains that make up the dextrin/Na-alginate/PVA hydrogel was responsible for the final stage of weight loss. The disintegration of the polymer chains themselves is indicated by this last stage of degradation, which releases smaller molecular fragments and breakdown products. The weight loss profiles that were observed during the thermal degradation analysis offer valuable insights into the intricate mechanisms and interactions involved in the degradation of the dextrin/Na-alginate/PVA hydrogel system. Notably, the degradation behavior of the hydrogel matrix is influenced by both the hydrogel composition and the presence of the drug molecule. The TGA of individual SA and PVA are depicted in Figs. S3–S4, respectively.

The article "Efficient drug delivery potential and antimicrobial activity of biocompatible hydrogels of dextrin/Na-alginate/PVA" was retracted in 2025. Reasons: unreliable results or conclusions; concerns about the authorship.

**Fig. 5:** Thermal analysis of the DSAPG#1 and drug loaded (CTX50) samples.

The dextrin/Na-alginate/PVA hydrogel sample was more stable in comparison to drug loaded hydrogel sample. The greater stability of the unloaded dextrin/Na-alginate/PVA hydrogel sample compared to the drug-loaded hydrogel sample could be due to several factors. The presence of the drug within the hydrogel matrix can introduce additional chemical interactions that may affect the stability of the hydrogel. These interactions could include drug-polymer interactions, drug-drug interactions, or changes in the crosslinking density of the hydrogel due to drug incorporation. The drug may not be fully compatible with the hydrogel matrix, leading to phase separation, aggregation, or other destabilizing effects. Incompatibility between the drug and the hydrogel components can compromise the structural integrity and stability of the hydrogel [38]. The presence of the drug within the hydrogel matrix may affect the swelling behavior of the hydrogel. Changes in swelling behavior can alter the physical properties of the hydrogel and potentially lead to decreased stability, especially if the drug induces excessive swelling or changes in the hydrogel structure. The drug-loaded hydrogel sample may exhibit accelerated degradation kinetics compared to the unloaded hydrogel sample. Drug molecules can accelerate hydrogel degradation by promoting chemical or enzymatic degradation pathways, leading to decreased stability over time. The drug-loaded hydrogel sample may require specific storage conditions (e.g., temperature, humidity) to maintain stability, whereas the unloaded hydrogel sample may be more stable under a wider range of storage conditions [4]. Hence, the presence of the drug within the hydrogel matrix introduces additional factors that can affect the stability of the hydrogel. These factors include chemical interactions, compatibility issues, changes in swelling behavior, degradation kinetics, and storage conditions, all of which can contribute to decreased stability compared to the unloaded hydrogel sample.

### 3.4 Swelling study

Swelling studies of unloaded DSAPG#1 with a crosslinker and DSAPG#2 (without a crosslinker) were compared (Fig. 6). It was observed that in the sample DSAPG#1, dextrin indicated a decreasing tendency of swelling versus time (min) in an acidic medium which exhibited its solubility in aqueous solution. This may occur because in an acidic medium, the protonation of hydrophilic groups occurs which inhibits the development of hydrogen bonding with water. At pH∼7.4, the swelling rate was increased because carboxylate ions of alginate got deprotonated which ionized the alginate and electrostatic repulsion occurred and allowed the hydrogel to absorb more water. Lower pH reduces broken carboxylic group in the alginate chain which in turn decreases the hydrophilicity. At pH∼7.4, the unloaded sample DSAPG#1 resulted in a higher swelling ratio [39]. In DSAPG#2, the swelling was less than the CTX50 at pH∼7.4, initially the swelling was increased and then a constant decrease was observed in the swelling ratio. Due to the presence of hydroxyl groups, PVA was hydrolyzed, which caused more ionization and resulted in creating spaces and enhanced the swelling ratio of the hydrogels [40]. The swelling trend exhibited the greater amount of dextrin in the blended sample is responsible for higher swelling versus the simple alginate-based sample [41]. The unloaded DSAPG#2 indicated a good swelling index as alginate and PVA give faster swelling due to loose packing and spaces in the structure of the hydrogel. At pH ∼7.4, besides dextrin, the –OH groups of PVA caused hydration with water as it is hydrophilic. As the density of blended hydrogels became greater, more acetal bonds were formed due to O–H groups. Therefore, hydrogen bonding between water-hydroxyl groups decreased, which decreased the hydrogel’s swelling. Hence, the unloaded DSAPG#1 (at pH ∼7.4) can be used for targeting drug delivery in a controlled way. The swelling ratio difference might be due to different compositions and components in the structure of hydrogel. The results indicated that an increase in the alginate ratio caused a decrease in the swelling ratio because an improvement in crosslink density caused water to hardly merge into the hydrogel structure [42]. Results also revealed that the loaded sample CTX50 exhibited better swelling than the CTX25.

The article "Efficient drug delivery potential and antimicrobial activity of biocompatible hydrogels of dextrin/Na-alginate/PVA" was retracted in 2025. Reasons: unreliable results or conclusions; concerns about the authorship.

**Fig. 6:** Swelling ratio of DSAPG#1, DSAPG#2, drug-loaded (CTX25 and CTX50) samples at pH 7.4.

### 3.5 Biodegradation behavior

Fig. 7 displays the results of a biodegradation test conducted on the prepared hydrogels in PBS solution. For the CTX50 sample, the weight loss on days 1, 3, and 6 was 26, 41, and 62 (%), respectively. While the biodegradation behavior of the other samples was similar, the biodegradation percentage of DSAPG#1, DSAPG#2, and CTX25 was lower than that of the CTX50 sample. The results of submerging the prepared hydrogels in phosphate-buffered saline (PBS) solution to assess their biodegradation are shown in Fig. 7. For example, on days 1, 3, and 6, the CTX50 sample showed weight loss of 26 %, 41 %, and 62 %, respectively. For the same duration, the biodegradation behavior of the other samples was similar. Remarkably, in comparison to the CTX50 sample, the DSAPG#1, DSAPG#2, and CTX25 samples showed a comparatively lower percentage of biodegradation. The different hydrogel formulations' varying rates of biodegradation point to potential variations in their structural makeup or crosslinking density, which may affect how susceptible they are to chemical or enzymatic breakdown in the PBS solution. These results show the possible influence of formulation parameters on the degradation behavior of the prepared hydrogels and offer insightful information about the biodegradation kinetics of the hydrogels. In-depth research into the fundamental processes causing these variations in biodegradation rates may aid in the creation of hydrogel formulations with customized degradation profiles for particular biomedical uses. Multiple factors can impact the hydrogel based on dextrin, Na-alginate, and PVA during its biodegradation process. The hydrogel's composition, specifically the proportions of PVA, Na-alginate, and dextrin, can influence how susceptible it is to biodegradation. Depending on their chemical structure and susceptibility to enzymatic or chemical degradation, different polymers may degrade at varying rates. The stability and resistance to degradation of the hydrogel network can be influenced by the extent of crosslinking present in it. Because higher crosslinking densities increase network stability, they usually lead to lower biodegradation rates. The rate and mode of biodegradation can be influenced by the hydrogel's physical characteristics, such as pore size and distribution. Greater interconnectivity and pore sizes may speed up degradation by making it simpler for degrading agents to reach polymer chains. There are several methods to characterize the biodegradation of dextrin/Na-alginate/PVA-based hydrogel, including weight loss measurements, morphological analysis, and evaluation of degradation products. Optimizing these hydrogels' performance in biomedical applications, like drug delivery, tissue engineering, and wound healing, requires an understanding of their biodegradation behavior.

**Fig. 7:** Biodegraadtion of DSAPG#1, DSAPG#2, drug loaded (CTX25 and CTX50) samples in PBS solution.

### 3.6 Drug release study and mechanism

After encapsulation of the drug, the release of the drug was examined in different media, i.e., PBS and SIF. The drug concentration was monitored by UV–visible analysis at 293 nm. The drug-loaded samples (CTX50 and CTX25 were immersed in 100 mL of PBS (pH∼7.4) and SIF (pH∼6.8) solutions at room temperature (37 °C). The mixture was stirred and at specific time intervals (10 min) 5 mL aliquots were withdrawn and 5 mL fresh (PBS and SIF) was added to prevent saturation of the drug. The drug release was monitored for 110 min. In the case of CTX25 in the SIF medium, the drug release was 18.6 % in the first 10 min, which increased linearly and reached 98.38 % in 70 min. Similarly, the CTX25 in PBS medium was recorded to be 12.4 % in the first 10 min, which reached 55.63 % in 60 min and the maximum drug release of CTX25 in PBS medium was 99.23 % at 110 min. From the data it is concluded that, drug release was fast initially and then declined with time. On the other hand, the CTX50 in the SIF medium revealed drug release of 15.3 % and 97.26 % after 10 and 80 min, respectively. In the case of PBS medium, the CTX50 released the drug at 11.63 % after 10 min, which reached 96.62 % after 110 min (Fig. 8). It was observed that the CTX drug release was fast in SIF media and case of PBS, the drug release was slow, which might be due the different nature of the media used for the drug release. From the data it is concluded that using hydrogel for the transfer of the drug, using *in-vitro* simulated intestinal fluid (SIF), the drug is easily absorbed from the intestine. The stimuli-responsive hydrogels can respond to external triggers such as temperature, light, or pH changes. These stimuli can be used to modulate drug release rates, providing on-demand or triggered release.

The article "Efficient drug delivery potential and antimicrobial activity of biocompatible hydrogels of dextrin/Na-alginate/PVA" was retracted in 2025. Reasons: unreliable results or conclusions; concerns about the authorship.

**Fig. 8:** The Ceftriaxone sodium release from the hydrogels (CTX25 and CTX50) in PBS and SIF media.

Multiple factors play a role in the mechanism of ceftriaxone sodium release from hydrogels based on dextrin, Na-alginate, and PVA. When water molecules come into contact with aqueous environments, the hydrogel matrix swells, enabling the water molecules to enter and interact with the polymer network. Pathways for the drug molecules to diffuse out of the hydrogel matrix are created by this swelling action. Concentration gradients cause the ceftriaxone sodium molecules to diffuse through the swollen hydrogel matrix. The size and charge of the drug molecules, as well as the hydrogel matrix's porosity and mesh size, all affect the rate of diffusion. The hydrogel's polymer matrix may degrade over time as a result of hydrolysis or enzymatic breakdown. The hydrogel matrix's integrity may be weakened by this breakdown process, which could result in the release of drug molecules that have been encapsulated [43].

The article "Efficient drug delivery potential and antimicrobial activity of biocompatible hydrogels of dextrin/Na-alginate/PVA" was retracted in 2025. Reasons: unreliable results or conclusions; concerns about the authorship.

Ion exchange processes within the hydrogel matrix can be aided by the presence of ions in the surrounding medium, such as sodium ions from Na-alginate. ceftriaxone sodium release can be affected by this ion exchange by changing the hydrogel's diffusivity and swelling behavior. Certain elements of the hydrogel matrix might have pH-sensitive characteristics, which would cause the swelling behavior and release kinetics to alter in response to pH changes. Under various physiological circumstances, the release of Ceftriaxone sodium can be modulated by this pH sensitivity. Overall, a complex mix of swelling, diffusion, polymer matrix degradation, ion exchange, and pH sensitivity processes are involved in the release of ceftriaxone sodium from hydrogels based on dextrin, Na-alginate, and PVA. The drug's release kinetics and behavior from the hydrogel matrix are determined by the combination of these factors [1,44,45].

Ceftriaxone sodium is a third-generation cephalosporin antibiotic used for the treatment of various bacterial infections by the parenteral route. Due to its slightly acidic nature, oral administration is not recommended. Different ratios of polyvinyl alcohol (PVA), sodium alginate (SA), dextrin (D) and glutaraldehyde (G) were used for the preparation of hydrogel and ceftriaxone sodium release. *In-vitro* simulated intestinal fluid (SIF) and phosphate-buffered saline (PBS) media were used for the drug release study and results are depicted in Fig. 8. Because according to international guidelines in drug development, any drug used by oral route, if it is released more than 10 % in simulated gastric fluid (SGF) initially in a half hour, those drugs are not considered for appropriate oral agent. In simulated intestinal fluid (SIF), ∼100 % drug (ceftriaxone sodium), loaded in hydrogel prepared by using different proportional ratios among polyvinyl alcohol (PVA), Sodium alginate (SA), dextrin (D) and glutaraldehyde (G) was released in 2 h. The developed hydrogels showed controlled release behavior in SIF and PBS media and hence, this drug can be delivered to the target to enhance its efficacy for biomedical applications.

These observations are in line with the previous reports and it was observed that the ceftriaxone sodium release from a hydrogel can be impacted by several variables, such as the drug's physicochemical characteristics, the hydrogel matrix's characteristics, and its surroundings. Drug diffusion, ion exchange, hydrogel swelling, polymer matrix degradation, pH sensitivity, and temperature sensitivity are some of the mechanisms underlying the release [27]. Ceftriaxone sodium release from a hydrogel is governed by several variables, including the hydrogel's composition, crosslinking density, and any controlled release modifications. Drug release profiles in particular hydrogel formulations must be understood and optimized through experimental research and thorough characterization. Hydrogels have the potential to provide controlled drug delivery, as shown by earlier research. To deliver ciprofloxacin hydrochloride, for instance Ref. [46], created a cross-linked hydrogel using dextrin and poly(2-hydroxyethyl methyl acrylate). Because of its slower rate of swelling and a higher percentage of crosslinking, the hydrogel demonstrated effective controlled release of the drug (36.78 % after 20 h), indicating that it is a promising matrix for drug loading and delivery. Similarly [47], blending pH-sensitive hydrogels using alginate, chitosan, and polyethylene glycol with crosslinker 1,4-diaminobutane via solution casting technique showed promise. Drug encapsulation and swelling ratio were studied in various solutions, including PBS, SGF, and SIF. The cumulative drug release profile of ceftriaxone sodium (CTX) indicated that the loaded hydrogels were optimal carriers for biomedical applications. Also [48], hydrogel films based on alginic acid, acrylic acid, and cyclodextrin were synthesized and characterized at various pH values. The hydrogels exhibited significant variations in properties, including kinetics release and drug encapsulating capacity. Hydrogel samples were synthesized at pH values of 1, 7, and 12. Ibuprofen drug delivery showed promise as pH-responsive for the hydrogels.

The article "Efficient drug delivery potential and antimicrobial activity of biocompatible hydrogels of dextrin/Na-alginate/PVA" was retracted in 2025. Reasons: unreliable results or conclusions; concerns about the authorship.

### 3.7 Antibacterial activity

Antibacterial activity of CTX25 and CTX50 (ceftriaxone sodium loaded) hydrogel samples, and control ciprofloxacin (1 mg/mL) were used against a panel of gram-positive and gram-negative microorganisms using agar well diffusion method to determine the biological effectiveness of the synthesized samples (Fig. 9) for the oral drug delivery of (ceftrixone sodium). The testing of loaded hydrogel sample was accomplished against a group of four bacteria including, *S. aureus, P. vulgaris, E. coli*, and *P. multocida*. Table 3 exhibited that in CTX50 (loaded sample), the significant zone of inhibition was observed by gram-negative bacteria *P. multocida* and gram-positive bacteria *S. aureus* [39]. The zones of inhibition in the case of CTX50 were found to be 16, 17, 16, and 17 (mm) against *P. vulgaris, S. aureus, E. coli,* and *P. multocida*, respectively and for CTX25, these values were 15, 12, 14, and 15 (mm), respectively. In the case of ciprofloxacin drug, the significant zone of inhibition was 19.3, 18.5, 19.67 and 20 (mm) against *P. vulgaris, S. aureus, E. coli,* and *P. multocida* strains, respectively. The antibacterial activity of CTX25 and CTX50 (ceftriaxone sodium loaded) hydrogel was comparable with the ciprofloxacin drug (1 mg/mL), which indicates the promising antibacterial potential of CTX25 and CTX50 blends.

The article "Efficient drug delivery potential and antimicrobial activity of biocompatible hydrogels of dextrin/Na-alginate/PVA" was retracted in 2025. Reasons: unreliable results or conclusions; concerns about the authorship.

**Fig. 9:** Antibacterial activity, zones of inhibition of drug-loaded membranes (CTX50 & CTX25) against a panel of microbial strains.

**Table 3:** Antibacterial activity (ZOI in mm) of membrane against gram-positive and gram-negative bacteria, using agar well diffusion method.

Sample code	P. vulgaris	S. aureus	E. coli	P. multocida
CTX50	16 ± 0.90	17 ± 1.30	16 ± 2.60	17 ± 0.90
CTX25	15 ± 2.40	12 ± 1.30	14 ± 3.10	15.3 ± 1.60
Standard	19.3 ± 1.20	18.5 ± 0.80	19.67 ± 1.20	20 ± 0.9

*E. coli: Escherichia coli: S. aureus: Staphylococcus aureus:, and P. multocida: Pasteurella multocida: P. vulgaris: Proteus vulgaris*. The values are mean ± SD of triplicate samples (n = 3); Standard = Ciprofloxacin (1 mg/mL).

Various processes are involved in the antibacterial activity mechanism of hydrogels based on dextrin, Na-alginate, and PVA that are loaded with ceftriaxone sodium. The broad-spectrum antibiotic ceftriaxone sodium is gradually released into the surrounding environment by the loaded hydrogel. By attaching to penicillin-binding proteins, breaking peptidoglycan cross-linking, and ultimately causing bacterial cell lysis, ceftriaxone sodium prevents the synthesis of bacterial cell walls. Via channels and pores in the bacterial cell membrane, released ceftriaxone sodium diffuses into the cell. Ceftriaxone sodium inhibits bacterial growth and causes cell death by interfering with vital cellular functions like protein synthesis, DNA replication, and cell wall formation once it has entered the bacterial cell [47]. Bacteria on the hydrogel's surface can interact directly with ceftriaxone sodium when it is released from the hydrogel. Bacterial cell wall are disrupted by this direct contact with the antibiotic, which eventually causes bacterial cell death and the leakage of cellular contents. The hydrogel's prolonged release of ceftriaxone sodium guarantees that bacterial cell are constantly exposed to the antibiotic, preserving its antibacterial efficacy for a considerable amount of time. The antibiotic's efficacy against bacterial growth and proliferation is bolstered by its sustained release profile [49]. Through synergistic effects, the combination of ceftriaxone sodium and the dextrin/Na-alginate/PVA hydrogel matrix may improve antibacterial activity. The hydrogel matrix might offer an environment that is favorable for the release and retention of antibiotics, enhancing ceftriaxone sodium's antibacterial activity. The dextrin/Na-alginate/PVA-based hydrogels loaded with ceftriaxone sodium exhibit an antibacterial activity mechanism that encompasses the following processes: the antibiotic is released gradually, diffuses into bacterial cells, kills surface bacteria upon contact, maintains antibacterial activity, and may have synergistic effects with the hydrogel matrix [50]. The antibacterial activity of hydrogels is critical, particularly in biomedical applications, where preventing or controlling bacterial infections is critical. The findings demonstrated that the synthesized hydrogels are a promising antibacterial agent, which is an important consideration for their potential biomedical applications.

The article "Efficient drug delivery potential and antimicrobial activity of biocompatible hydrogels of dextrin/Na-alginate/PVA" was retracted in 2025. Reasons: unreliable results or conclusions; concerns about the authorship.

### 3.8 Cytotoxicity analysis

For analyzing the *in-vitro* cytotoxicity of hydrogel, cultured cells are usually subjected to extracts or direct contact with the hydrogel material, and their viability, morphology, and metabolic activity are evaluated. This analysis offers important information for biomedical applications and aids in assessing the hydrogel's possible cytotoxic effects on cells. Prepared specimens were examined with isolated RBCs (young volunteers) to test the stability of the erythrocyte cell membrane. The process is simple and *in vitro* for precursory screening afterward it proceeds towards further animal study and results are presented in Table 4. A sterile chilled, phosphate buffer saline (pH∼7.4) was used as the negative control (0 % background RBCs cell lysis) and Triton X-100 (0.1 %) was used as a positive control (100 % RBCs cell lysis). The CTX50 and CTX25 showed 9.75 and 9.42 (%) RBCs lysis, which indicates that the prepared hydrogels are nontoxic as it is observed in *in-vitro* cytotoxicity analysis against RBCs. The ability of a substance to harm or kill cells is referred to as cytotoxicity. Cytotoxicity analysis is an important consideration in the context of drugs, particularly in the development of agents used for drug delivery. Cytotoxic drugs can harm the body cells, potentially leading to side effects. In this context, the hydrogels are safer and suitable for Ceftriaxone sodium drug delivery.

**Table 4:** Cytotoxicity (%) analysis of drug-loaded hydrogel against red blood cells (RBCs).

Sr.#	Sample code	**RBCs lysis (%)**
1	CTX50	7.75 ± 2.57
2	CTX25	7.42 ± 3.59
3	PBS (Negative control)	0 %
4	Triton-x100 (0.1 %) (Positive control)	100 %

Cytotoxicity analysis is a useful tool for predicting the biocompatibility of hydrogel materials in-vivo by offering important insights into the possible negative effects of these materials on mammalian cells. It enables scientists to evaluate the hydrogel's safety for use in scaffolds for tissue engineering, medication delivery systems, and medical devices. Quantitative assessments of cell viability are obtained through cytotoxicity assays. This makes it possible to evaluate the hydrogel's cytotoxic effects accurately and consistently, and it makes comparing formulations and concentrations easier [2]. The hydrogel extract can be used in cytotoxicity assays at low concentrations to identify minute alterations in cell viability because of their high sensitivity. The detection of possible cytotoxic effects is made possible by this sensitivity. It's simple to modify cytotoxicity assays for high throughput screening of various hydrogel conditions or formulations. This makes it possible to quickly and effectively sort through huge libraries of hydrogel materials to find the ones with the best biocompatibility profiles. Cultured mammalian cells can be used to perform cytotoxicity analysis, removing the need for animal testing and addressing ethical issues related to *in-vivo* research [1]. The 3Rs (Replacement, Reduction, Refinement) in animal research are in line with this methodology. Cytotoxicity analysis is a typical part of the biocompatibility testing that regulatory bodies need to conduct to approve pharmaceuticals and medical devices. Researchers can ensure regulatory compliance and expedite the transition of hydrogel-based therapies to clinical applications by conducting cytotoxicity analyses [45]. Hence, cytotoxicity analysis of dextrin/Na-alginate/PVA-based hydrogels loaded with ceftriaxone sodium provides a strong and trustworthy approach for evaluating their safety and biocompatibility, aiding in the creation of secure and efficient biomedical products.

The article "Efficient drug delivery potential and antimicrobial activity of biocompatible hydrogels of dextrin/Na-alginate/PVA" was retracted in 2025. Reasons: unreliable results or conclusions; concerns about the authorship.

## 4 Conclusion

A biocompatible hydrogel for targeted drug delivery applications was prepared based on dextrin, alginate, and PVA. The hydrogels were characterized to determine the effect of different combinations of natural polymers (dextrin and alginate) and synthetic polymers (PVA) on the properties of the hydrogel. The hydrogels (DSAPG#1 and DSAPG#2) demonstrated promising properties, including swelling, biodegradation, morphology, antimicrobial activity and drug release efficiency. These findings suggest that this hydrogel has promising efficiency for the loading and release of ceftriaxone sodium. The ceftriaxone sodium-loaded hydrogel demonstrated an effective drug release rate at pH ∼7.4. The surface morphology was significantly changed in hydrogels in response to drug loading. The hydrogels showed promising antibacterial activity against a panel of gram-positive and gram-negative bacterial strains. Furthermore, the cytotoxicity study revealed the nontoxic nature of the prepared hydrogel, confirming the effectiveness and safety of the prepared sample for potential biomedical applications. This comprehensive study emphasizes the developed hydrogel's promising properties, emphasizing its potential utility in targeted drug delivery and biomedical applications. Preclinical and clinical investigations to assess the safety and effectiveness of the created hydrogel in animal models, could be the main focus of future research. Evaluating the hydrogel formulation's shelf life and long-term stability ensures it is viable for real-world biomedical applications. The hydrogel's eventual clinical translation depends on its scalability and the availability of feasible manufacturing techniques for large-scale production.

The article "Efficient drug delivery potential and antimicrobial activity of biocompatible hydrogels of dextrin/Na-alginate/PVA" was retracted in 2025. Reasons: unreliable results or conclusions; concerns about the authorship.

## Funding

This research was funded by Princess Nourah bint Abdulrahman University Researchers Supporting Project number (PNURSP2024R488), Princess Nourah bint Abdulrahman University, Riyadh, Saudi Arabia.

## Data availability statement

Data will be made available on request.

## CRediT authorship contribution statement

**Arif Nazir:** Supervision. **Mazhar Abbas:** Project administration, Methodology. **Faiza Kainat:** Writing – original draft, Investigation. **Dure Najaf Iqbal:** Conceptualization. **Farheen Aslam:** Data curation. **Abida Kamal:** Formal analysis. **Osama A. Mohammed:** Validation, Software, Investigation. **Kinza Zafar:** Writing – original draft, Investigation. **Amal Abdullah Alrashidi:** Validation, Resources, Formal analysis. **Samar Z. Alshawwa:** Validation, Resources, Funding acquisition. **Munawar Iqbal:** Writing – review & editing, Visualization.

## Declaration of competing interest

The authors declare that they have no known competing financial interests or personal relationships that could have appeared to influence the work reported in this paper.
